# NGF protects neuroblastoma cells against β‐amyloid‐induced apoptosis via the Nrf2/HO‐1 pathway

**DOI:** 10.1002/2211-5463.12742

**Published:** 2019-11-01

**Authors:** Rui Su, Wei Su, Qian Jiao

**Affiliations:** ^1^ Department of Neurosurgery Luoyang Central Hospital Affiliated to Zhengzhou University China; ^2^ Department of Intensive Care Unit Sir Run Run Shaw Hospital Affiliated by Zhejiang University School of Medicine Hangzhou China; ^3^ Department of Anesthesia Surgery Sanmenxia Central Hospital China

**Keywords:** apoptosis, JNK/c‐Jun, NGF, Nrf2, β‐amyloid

## Abstract

As one of the main neurotrophic factors, nerve growth factor (NGF) participates in various processes related to viability, plasticity, and neuronal growth. NGF is known to protect against cell death and toxicity triggered by β‐amyloid (Aβ), but the underlying mechanism remains unclear. Here, we investigated this process in SKNSH neuroblastoma, in which NGF reduced cell death induced by Aβ25–35. Furthermore, NGF suppressed the production of reactive oxygen species (ROS) and promoted antioxidant function via Aβ25–35. Additionally, we demonstrated that NGF impaired the activation of the JNK/c‐Jun signaling pathway and significantly increased Nrf2 nuclear translocation and HO‐1 expression. Nrf2 elimination abolished the protective effect of NGF‐1 on Aβ25–35‐induced ROS generation, apoptosis, and activation of the JNK/c‐Jun pathway. The results of our study indicate that NGF protects neuroblastoma against injury triggered by Aβ25–35 via suppression of ROS–JNK/c‐Jun pathway stimulation through the Nrf2/HO‐1 pathway.

## Abstract 2

Nerve growth factor (NGF) promotes the nuclear translocation of Nrf2 and subsequently upregulates HO‐1 expression. This reduces the levels of reactive oxygen species (ROS), which attenuates the activation of JNK/c‐Jun pathway and eventually contributes to deceased cell apoptosis. The present discovery of this novel NGF/Nrf2/HO‐1 pathway and ROS–JNK/c‐Jun pathway identifies new clinical targets for therapeutic intervention of Alzheimer's disease.

**Abbreviations**
AD: Alzheimer's disease
Aβ: β‐amyloid
CAT: catalase
CNS: central nervous system
ER: endoplasmic reticulum
FC: flow cytometry
NFTs: neurofibrillary tangles
NGF: nerve growth factor
OS: oxidative stress
PNS: peripheral nervous system
ROS: reactive oxygen species
SOD: superoxide dismutase

As the most prevalent neurodegenerative disease, Alzheimer's disease (AD) is characterized by the occurrence of senile plaques (mainly filled with Aβ assemblies); malfunction of synapses; intracellular neurofibrillary tangles (NFTs), including hyperphosphorylated tau proteins; and loss of dystrophic neurites and neurons 1, 2. Despite the fact that various approaches have been studied in order to decrease the incidence of AD, almost no advancements have been made. Several mechanisms, such as neurotrophic injury and cell death, participate in AD development 3, 4. It has been previously reported that the apoptosis of neurons in AD is mainly triggered by Aβ 5, 6. The understanding of cell death triggered by Aβ remains insufficient, but previous studies have indicated that oxidative stress (OS) participates in the reaction 7. Increasing evidence suggests that OS is regarded as executor of neuronal toxicity triggered by Aβ and participates in AD generation 8, 9. Promoted oxidation of proteins, DNA, and lipids has been discovered in AD brains 10. Furthermore, elevated concentrations of OS markers in the blood of AD mice have been shown to exist prior to the generation of plaques 11. Consequently, modulating brain OS may be promising in the treatment of AD.

As a part of the neurotrophin group, nerve growth factor (NGF) is a type of growth factor that has been widely investigated 12. Previous studies have revealed that NGF participates in the viability, development, and preservation of neurons in mammalian nervous systems 13, 14. For example, NGF affects the development of sensory neurons arising from the neural crest in the peripheral nervous system (PNS), cholinergic neuronal cells of the central nervous system (CNS), and sympathetic neurons 15. In addition to neuronal cells, NGF expression has been found in several types of glial cells, including olfactory ensheathing cells, microglial cells, oligodendrocytes, and astrocytes 16, 17. Recent studies have shown that NGF leads to neuronal viability and apoptosis in aging, and neurodegenerative distress 18, 19. It has been recently reported that NGF is linked to the pathogenesis, etiology, and clinical manifestations of AD 20. Elimination of NGF in adult murine models via expression of transgenic anti‐NGF antibodies led to the decline in cholinergic neuronal cells in the hippocampus and basal forebrain 21. NGF elimination in murine models has also been shown to lead to pathogenesis similar to that of AD, for example, the aggregation of Aβ, hyperphosphorylation of tau, and malfunction of synapses. Supplementation with NGF promotes alterations in the pathology of Aβ and suppresses memory damage in AD mice 22, 23. This evidence indicates that NGF is able to serve as a reliable suppressor of cell toxicity triggered by Aβ. Nevertheless, the understanding of its mechanism is still insufficient. Our study aimed to investigate how NGF defends against cell death in SKNSH cells. Our results demonstrate that the Nrf2–ROS–JNK pathway modulates the influence of NGF on cell death triggered by Aβ, emphasizing that NGF may be promising for future AD therapies.

## Materials and methods

### Cell culture and treatment

SKNSH cells were obtained from ATCC (American Type Culture Collection, Manassas, VA, USA). DMEM (Gibco, Gaithersburg, MD, USA) was applied to cell cultivations in 5% CO_2_ at 37 °C. Double‐distilled water was used to dissolve the Aβ25–35 (Sigma, St Louis, MO, USA). For aggregation, incubation lasting seven to ten days was carried out at 37 °C. A series of concentrations (0, 5, 10, 25, and 50 μm) of Aβ25–35 were added to the cultures after aggregation in order to trigger oxidative insult. Medium without serum was applied to the cells for 6, 12, 24, or 48 h. Preliminary incubation with NGF (0, 25, 50, 100, or 200 ng·mL^−1^; Cell Signaling Technology, Boston, MA, USA) was carried out 24 h prior to supplementing the cultures with Aβ25–35. This study has been approved by the Ethics Committee of Luoyang Central Hospital Affiliated to Zhengzhou University.

### primary neurons cultures

primary neurons cultures were prepared from the cortical tissues of C57BL/6 mice on embryonic day 14/15 (E14/15). Cells were plated at 0.9 × 10^6^ per well (12‐well plate) on poly‐d‐lysine‐ and laminin‐coated glass coverslips. Cells were grown in Basal Medium Eagle (all media supplied from Gibco, Rockville, MD, USA) supplemented with in Neurobasal Media supplemented with 2% B27. All animal procedures were performed in strict accordance with the guideline of the Institutional Animal Care and Use Committee (IACUC) of Luoyang Central Hospital Affiliated to Zhengzhou University.

### Evaluation of cell survival

Evaluation of cell survival was carried out using a CCK‐8 assay. At the preliminary time point determined prior to termination of treatment, CCK‐8 (100 μL) was added to every well. The absorbance under 450 nm was detected using a multiwell spectrophotometer (Bio‐Rad, Hercules, CA, USA).

### Flow cytometry

Cold phosphate‐buffered saline was used to wash the cells twice. The supernatant was then eliminated subsequent to a 5‐min centrifugation at 1000 *g*. Binding buffer was added to the resuspension. FITC–Annexin V and propidium iodide (PI) were added according to the manufacturer’s instructions. A FACScan flow cytometer (Becton, Dickinson and Company, Franklin Lakes, NJ, USA) was used to evaluate fluorescence signals.

### Measurement of intracellular ROS

The fluorescent probe CM‐H2DCFDA, which is specific to reactive oxygen species (ROS), was used to evaluate intracellular ROS. A 30‐min incubation was carried out using 25 μm H2DCFDA. PBS was used to wash the cells twice. Multiwell spectrophotometry was used to conduct fluorescence assessment. The ROS generation intensity of the cells in the control group was manually determined to be 100%.

### Measurement of superoxide dismutase and catalase function

Catalase (CAT) and superoxide dismutase (SOD) functions were measured by colorimetric assay kit (Abcam, Cambridge, MA, USA). In short, a lysis buffer was applied for protein separation. The protein extract (10 μg) was applied to the antioxidant enzymes. A multiwell spectrophotometer was used to evaluate the absorbance for SOD (450 nm) and CAT (520 nm).

### siRNA and cell transfection

Transfection of Nrf2 siRNA oligoribonucleotide (50 nm; Santa Cruz Biotechnology, Santa Cruz, CA, USA) was carried out using RNAiFect transfection reagent (Qiagen, Inc., Shanghai, China). The negative sequence of siRNA served as a control. Cells received an extra 24‐h incubation in medium with 0.5% serum prior to activation.

### Western blot

Lysis buffer (Beyotime, Wuhan, China) was applied to homogenize the lysates. Bradford assay (Bio‐Rad) was used for protein quantification. SDS/PAGE was carried out for protein evaluation. Protein isolation was carried out using 8–15% Tris/HCl polyacrylamide gels (Bio‐Rad) before transferring the proteins to a PVDF membrane (Millipore, Bedford, MA, USA). Subsequent to blocking, overnight incubation was conducted at 4 °C with the primary antibodies (anti‐c‐Jun, anti‐phospho‐c‐Jun, anti‐JNK, anti‐phospho‐JNK, anti‐Nrf2, anti‐H3, anti‐PUMA, anti‐β‐actin, and anti‐HO‐1) before adding the secondary HRP‐conjugated antibodies.

### Statistical analysis

Results are presented as mean ± SEM. Differences were evaluated using ANOVA with Tukey’s post hoc analysis. Results were regarded as significant at a *P* value < 0.05.

## Results

### NGF reduced Aβ25–35‐triggered neuronal toxicity in SKNSH cells

Neuronal toxicity of SKNSH cells was determined by a CCK‐8 assay subsequent to incubation with different concentrations and application times of Aβ25–35. Aβ25–35 significantly increased apoptosis (Fig. 1A,B). Cell survival after supplementation with NGF (25, 50, or 100 ng·mL^−1^) was similar to that in the control group. However, NGF at a concentration of 200 ng·mL^−1^ brought about a noticeable decline in survival (Fig. 1C). In order to explore the influence of NGF on neuronal toxicity, SKNSH cells received Aβ25–35 with or without NGF for 24 h. Stimulation of SKNSH cells with Aβ25–35 led to a significant decrease in cell viability after 24 h. Treatment with NGF suppressed Aβ25–35‐induced cytotoxicity (Fig. 1D). The protective role of NGF was also confirmed in primary neurons (Fig. 1E). These findings demonstrate that NGF ameliorated the neuronal toxicity triggered by Aβ25–35 in SKNSH cells.

**Figure 1:** NGF defends against Aβ25–35‐triggered neuronal toxicity in SKNSH cells. (A) Twenty‐four‐hour incubation was conducted using various Aβ25–35 concentrations. Scale bars: 100 nm. (B) Cells received supplementation with Aβ25–35 (25 μm) for the indicated time. (C) Cells received supplementation with NGF at the particular concentrations for 24 h. (D, E) Cells received preliminary NGF supplementation (0, 25, 50, or 100 ng·mL^−1^) for 24 h before the addition of 25 μm Aβ25–35. Survival was evaluated using a CCK‐8 assay in SKNSH cells (D) and primary neurons (E). Results are expressed as mean ± SEM for three independent experiments. One‐way ANOVA, *P < 0.05, **P < 0.01 vs. control; ^#^ *P* < 0.05, ^##^ *P* < 0.01 vs. Aβ25–35 alone.

### NGF suppressed cell apoptosis triggered by Aβ25–35 in SKNSH cells

In order to evaluate the influence of NGF on cell apoptosis triggered by Aβ25–35, dual staining with Annexin V–FITC and PI was used to evaluate apoptosis via flow cytometry (FC). NGF (100 ng·mL^−1^) alone did not influence the death of SKNSH cells (Fig. 2A,B). Supplementing with Aβ25–35 led to a noticeable promotion in the proportion of apoptosis after 24 h. NGF noticeably suppressed Aβ25–35‐triggered promotion of cell death from 31.2 ± 2.87% to 10.1 ± 1.01%. In addition, NGF significantly suppressed Aβ25–35‐triggered apoptosis in primary neurons (Fig. 2C). These findings suggest that NGF inhibited the apoptosis of SKNSH cells triggered by Aβ25–35.

**Figure 2:** NGF reduced Aβ25–35‐triggered cell apoptosis in SKNSH cells. SKNSH cells received preliminary supplementation with NGF (100 ng·mL^−1^) for 24 h prior to a 24‐h treatment with Aβ25–35 (25 μm). (A) Representative apoptosis depicted by FC. (B, C) Quantification of cell apoptosis in SKNSH cells (B) and primary neurons (C). Results are expressed as mean ± SEM for three independent experiments. One‐way ANOVA, **P < 0.01 vs. control; ^#^ *P* < 0.05 vs. Aβ25–35 alone.

### NGF inhibited Aβ25–35‐induced JNK/c‐Jun signal pathway activation in SKNSH cells

Previous studies have revealed that JNK/c‐Jun activation participates in the cell death of neurons triggered by Aβ 23. Nevertheless, the mechanism by which the JNK/c‐Jun pathway correlates with the defensive influence of NGF is unclear. In our study, western blot was used to evaluate JNK/c‐Jun expression. Aβ25–35 was found to promote JNK and c‐Jun phosphorylation as well as the expression of the pro‐apoptotic protein PUMA. NGF remarkably suppressed the promotion of PUMA expression as well as the phosphorylation of JNK/c‐Jun triggered by Aβ25–35 (Fig. 3). These findings suggest that NGF inhibited the cell death triggered by Aβ25–35 via suppression of JNK/c‐Jun pathway activation in SKNSH cells.

**Figure 3:** NGF suppressed Aβ25–35‐triggered JNK/c‐Jun activation in SKNSH cells. SKNSH cells received preliminary supplementation with NGF (100 ng·mL^−1^) for 24 h prior to 24‐h stimulation with Aβ25–35 (25 μm). (A–D) Representative immunoblots (A) and quantitative evaluation of p‐JNK (B), p‐c‐Jun (C), and PUMA (D) in SKNSH cells. Results are expressed as mean ± SEM for three independent experiments. One‐way ANOVA, **P < 0.01 vs. control; ^#^ *P* < 0.05 vs. Aβ25–35 alone.

### NGF ameliorated ROS production triggered by Aβ25–35 in SKNSH cells

ROS serves as a promising mechanism for neuronal death triggered by Aβ 24. In order to better determine the influence of NGF, we evaluated ROS levels in the cells using an H2DCFDA assay. NGF remarkably inhibited the ROS generation triggered by Aβ25–35 that was measured via H2DCFDA fluorescence (Fig. 4A). CAT and SOD served as essential antioxidant enzymes. Supplementing with Aβ25–35 led to a decline in the functions of both CAT and SOD. On the contrary, preliminary supplementation with NGF restored the declining enzyme function of CAT and SOD that was triggered by Aβ25–35 (Fig. 4B,C). In addition, NGF significantly reduced the ROS level in primary neurons (Fig. 4D). These findings suggest that NGF ameliorated the production of ROS triggered by Aβ25–35 in SKNSH cells.

**Figure 4:** NGF ameliorated ROS production triggered by Aβ25–35 in SKNSH cells. SKNSH cells received preliminary NGF supplement (100 ng·mL^−1^) for 24 h prior to 24‐h treatment with Aβ25–35 (25 μm). A. Intracellular ROS was measured via oxidation of H2DCFDA to DCF in SKNSH cells. B. Superoxide dismutase activity was measured using a colorimetric assay kit. C. A catalase‐specific activity assay kit was used to measure CAT function. D. A. Intracellular ROS was measured via oxidation of H2DCFDA to DCF in primary neurons. Results are expressed as mean ± SEM for three independent experiments. One‐way ANOVA, ^*^ *P* < 0.05, ^**^ *P* < 0.01 vs. control; ^#^ *P* < 0.05 vs. Aβ25–35 alone.

### NGF promotes Nrf2/HO‐1 expression in SKNSH cells

It has previously been shown that Nrf2/HO‐1 is essential to the resistance of neurons to OS triggered by Aβ 25. In order to explore the influence of the Nrf2/HO‐1 pathway in the defensive effect modulated by NGF in SKNSH cells, our research investigated Nrf2/HO‐1 expression in SKNSH cells subsequent to supplementation with NGF. Our results show that the nuclear Nrf2 concentration was significantly elevated and that the cytoplasmic Nrf2 concentration noticeably declined subsequent to NGF supplementation (Fig. 5A–C), suggesting that NGF increased Nrf2 nuclear translocation. Additionally, NGF promoted the downstream expression of HO‐1 (Fig. 5D). These findings indicate that the Nrf2/HO‐1 signaling pathway may participate in the defensive influence of NGF in SKNSH cells.

**Figure 5:** Nerve growth factor promotes Nrf2/HO‐1 expression in SKNSH cells. SKNSH cells received NGF supplement (100 ng·mL^−1^) for 24 h. (A–D) Representative immunoblots (A) and quantitative evaluation of nuclear (n) Nrf2 (B), cytoplasmic (c) Nrf2 (C), and HO‐1 (D) in SKNSH cells. Results are expressed as mean ± SEM for three independent experiments. One‐way ANOVA, *P < 0.05, **P < 0.01 vs. control.

### Nrf2/HO‐1 is necessary for the protective effects of NGF against apoptosis induced by Aβ25–35 in SKNSH cells

In order to better investigate the influence of the Nrf2/HO‐1 signaling pathway on the defensive effects of NGF, we inhibited the expression of Nrf2 in SKNSH cells using Nrf2‐specific siRNA (Fig. 6A,B). As shown in Fig. 6C, NGF suppressed the apoptosis triggered by Aβ25–35 that was attenuated via Nrf2 elimination. Furthermore, Nrf2 deficiency eliminated the suppressive influence of NGF on the generation of ROS (Fig. 6D). NGF suppressed JNK/c‐Jun activation by decreasing JNK/c‐Jun phosphorylation as well as by decreasing the expression of PUMA. Nrf2 knockdown abrogated the suppressive influence of NGF on JNK/c‐Jun stimulation (Fig. 6E–H). These findings demonstrate that the defensive influence of NGF against cell death triggered by Aβ25–35 is based on the Nrf2/HO‐1 signaling pathway.

**Figure 6:** Nrf2/HO‐1 mediated defensive influence of NGF against apoptosis triggered by Aβ25–35 in SKNSH cells. Twenty‐four‐hour transfection of SKNSH cells was carried out with Nrf2 siRNA and subsequently supplemented with Aβ25–35 or Aβ25–35 + NGF for 24 h. (A, B) Representative immunoblots (A) and quantitative evaluation of Nrf2 (B) in SKNSH cells. (C) FC was used for the assessment of cell death. (D) Intracellular ROS was evaluated via the oxidation of H2DCFDA to DCF. (E–H) Representative immunoblots (E) and quantitative evaluation of p‐JNK (F), p‐c‐Jun (G), and PUMA (H) in SKNSH cells. Results are expressed as mean ± SEM for three independent experiments. Two‐way ANOVA, **P < 0.01 vs. control; ^#^ *P* < 0.05 vs. Aβ25–35 alone; ^$^ *P* < 0.05 vs. Aβ25–35+NGF.

## Discussion

The Nrf2/HO‐1 signaling pathway mediates a defensive influence of NGF in SKNSH cells against apoptosis triggered by Aβ25–35. NGF promotes Nrf2/HO‐1 expression, which decreases ROS concentration, inhibits JNK/c‐Jun stimulation, and ultimately contributes to a suppressive influence on the apoptosis triggered by Aβ25–35.

Nerve growth factor displays neuronal protective and refreshing influences in the CNS 26. Previous studies have shown that NGF decreases mitochondrial and nuclear apoptosis and increases the differentiation and viability of neurons by stimulating ERK and PI3K 27. It has recently been shown that NGF decreases the death of Schwann cells and endoplasmic reticulum (ER) stress triggered by high concentrations of glucose 28. NGF downregulates the phosphorylation of APP at the neuron‐specific residue T668, promotes APP binding with TrkA, and favors APP trafficking to the Golgi, at the expense of BACE interaction and cleavage. In our study, we demonstrated that NGF suppressed the death of SKNSH cells triggered by Aβ25–35. It has been reported that JNK/c‐Jun is stimulated in AD neurons and is essential to the neuronal apoptosis triggered by Aβ in animal models of AD 29. JNK function is promoted in the cortex and essential to the pathology of AD, including the accumulation of amyloid, hyperphosphorylation of tau protein, and the malfunction of synapses in AD mice 30, 31. Expression of c‐Jun is downregulated by siRNA and suppresses apoptosis in the hippocampus and cortex in reaction to Aβ 32. Previous studies have demonstrated that c‐Jun is able to increase the cell death of sympathetic neuronal cells subsequent to NGF removal, and of neuronal cells in the cortex in reaction to the toxicity of arsenite and injury to DNA. The function of c‐Jun can be downregulated via neutralizing antibody, conditional gene deletion, or dominant‐negative construct, or through mutant construct lacking stimulation phosphorylation locations. Death of sympathetic neurons is inhibited by c‐Jun downregulation subsequent to NGF elimination 33. In our study, it was shown that NGF was able to inhibit the stimulation of phosphorylation and the decreased expression of PUMA. Various studies suggest that PUMA is a promising means to increase cell death that may be directly aimed at JNK/c‐Jun 32. In summary, the findings of our study indicate that NGF defends against the cell death triggered by Aβ through JNK/c‐Jun suppression.

It has been shown that ROS participates in AD pathology as well as the neuronal toxicity of Aβ 34. A number of studies have suggested that Aβ and OS are correlated with one another since OS is triggered by Aβ accumulation *in vitro* and *in vivo*. Oxidative products and agents increase the expression of APP and Aβ concentration in neuronal and other cells 35. Extra aggregation of ROS has been shown to cause DNA injury and trigger the peroxidation of lipids, ultimately causing apoptosis 8. It is widely accepted that ROS serves as an essential regulator in various pathways such as JNK 36. Our study demonstrated that supplementation with Aβ25–35 led to a remarkable elevation in ROS generation inside the cells as well as a noticeable decline in the functions of CAT and SOD, similar to previous studies. ROS concentration inside the cells was suppressed by NGF, which then suppressed JNK/c‐Jun activation. These findings indicate that NGF inhibits the cell death triggered by Aβ via ROS–JNK/c‐Jun suppression.

Nrf2 modulates antioxidant agents that defend against oxidative injury induced by multiple types of damage as well as inflammation 37. Under normal circumstances, Nrf2 is located in the cytoplasm in an inactive form that results from Keap1 binding. As soon as Nrf2 is stimulated, nuclear translocation occurs. Nrf2 triggers antioxidative transcription of SOD, HO‐1, and CAT 38. In our study, it was demonstrated that NGF increased Nrf2 nuclear translocation and elevated the expression of HO‐1. NGF decreased ROS concentration, which impaired JNK/c‐Jun stimulation and caused cell apoptosis (Fig. 7). Nrf2 knockdown eliminated the defensive influence of NGF on ROS production, JNK/c‐Jun stimulation, and cell death triggered by Aβ. The findings of our study suggest that Nrf2/HO‐1 is essential to the defensive influence of NGF against the death of SKNSH cells triggered by Aβ25–35.

**Figure 7:** Schematic layout depicting that NGF defends neuroblastoma against cell death triggered by Aβ25–35 via suppression of ROS–JNK/c‐Jun pathway activation through the Nrf2/HO‐1 pathway. NGF increases Nrf2 nuclear translocation and promotes expression of HO‐1. NGF decreases ROS concentration, which impairs the stimulation of the JNK/c‐Jun signaling pathway and results in a decrease in apoptosis.

## Conclusions

In conclusion, our research shows that NGF defends neuroblastoma against the cell death triggered by Aβ25–35 via ROS–JNK/c‐Jun suppression through the Nrf2/HO‐1 pathway. Our findings provide innovative targets for the treatment of AD.

## Conflict of interest

The authors declare no conflict of interest.

## Author contributions

RS and QJ conceived and designed the project and wrote the paper, WS acquired the data, and RS and WS analyzed and interpreted the data.
